This article has been retracted.

# Stellate Ganglion Block Combined with Dexmedetomidine Protects Obese Rats from Lipopolysaccharide-Induced Acute Lung Injury

**DOI:** 10.1155/2022/5635063

**Published:** 2022-03-29

**Authors:** Weiwei Zhang, Pengfei Li, Xiang Gao, Zhigan Lv

**Affiliations:** ^1^Department of Anesthesiology, Shanxi Bethune Hospital, Shanxi Academy of Medical Sciences, Tongji Shanxi Hospital, Third Hospital of Shanxi Medical University, Taiyuan 030032, China; ^2^Department of Anesthesiology, Tongji Hospital, Tongji Medical College, Huazhong University of Science and Technology, Wuhan 430030, China; ^3^Translational Medicine Research Center, Shanxi Medical University, Taiyuan, China; ^4^Department of Pain Treatment, Shanxi Bethune Hospital, Shanxi Academy of Medical Sciences, Tongji Shanxi Hospital, Third Hospital of Shanxi Medical University, Taiyuan 030032, China

## Abstract

**Objective:**

To investigate the effect and mechanism of combined stellate ganglion block (SGB) and dexmedetomidine (Dex) in obesity-related acute lung injury.

**Methods:**

Thirty-six 4-week-old male Wistar rats were randomly divided into 6 groups, each with 6 rats: blank group (Control), high-fat diet group (HFD), high-fat + lipopolysaccharide (LPS)-induced acute lung injury group (HFD + LPS), SGB group, Dex group, and SGB + Dex group. H&E staining detected the pathological structure of rat lung tissue. TUNEL staining was used to examine cell apoptosis in lung tissue. Oxidative factors were accessed by biochemical reagents. ELISA was employed to measure the levels of TNF-*α*, IL-1*β*, and MCP1 in rat alveolar lavage fluid. Western blot detected the protein expression of glucose-regulated Protein 78 (GRP78), C/EBP homologous protein (CHOP), protein kinase R-like endoplasmic reticulum kinase (PERK), and p-PERK in lung tissue.

**Results:**

The body weight of rats in the HFD group was higher than that in the control group. The use of SGB or Dex alone could significantly reduce the rate of pulmonary edema and lung cell apoptosis in HFD-induced obese rats and reduce MPO, TNF-*α*, IL-1*β*, and MCP1 levels, increasing the activity of SOD and GSH-Px. In addition, using SGB or Dex alone can also significantly reduce the protein expression levels of GRP78, CHOP, and p-PERK. The combined use of SGB and Dex can enhance the above effects.

**Conclusion:**

The combined use of SGB and Dex can protect against obesity-related acute lung injury and is more effective than using SGB or Dex alone.

## 1. Introduction

Acute lung injury (ALI) is a type of respiratory disease caused by a variety of intrapulmonary and extrapulmonary triggers, which is mainly characterized by respiratory distress, hypoxemia, chronic persistent inflammatory response, and non-cardiogenic pulmonary edema caused by increased vascular permeability [1]. In recent years, due to air pollution and changes in human living habits, the incidence of ALI/ARDS has increased day by day. Over 600 million adults worldwide are suffering from obesity [2]. Epidemiological studies have shown that obesity is an important predisposing factor in the pathogenesis onset of ALI [3]. At present, the main clinical treatment strategies include the treatment of the primary disease, respiratory support, sedative treatment, circulatory function support, etc., but there is no specific medicine for the treatment of ALI.

Dexmedetomidine (Dex), as a highly effective and highly selective *α*2 adrenergic receptor agonist, is widely used in clinical surgical anesthesia and ICU sedation due to its good analgesic, sedative, and anti-sympathetic effects [4]. The anti-sympathetic effect of Dex can also weaken the stress response and reduce the secretion of stress hormones such as cortisol [5]. In recent years, with more and more in-depth research on Dex, it has been found that it has a protective effect on organ damage. Studies have indicated that Dex attenuates the inflammatory response associated with sepsis via central alpha 2A adrenergic receptors. In addition, Dex exerts a protective effect by reducing inflammatory responses on various organs such as the nervous system, heart, lungs, kidneys, liver, and small intestine [6, 7]. Dex has been proven to suppress the inflammatory response and prevent multiple organ damage under various conditions and can reduce ALI caused by heatstroke (HS). However, in clinical use, it was found that Dex did not improve mortality and ventilator-free days, and its treatment of ALI was limited [8]. Therefore, there is an urgent need for effective drugs to improve the efficacy of Dex.

Stellate ganglion (SG) is formed by the fusion of cervical 6 and 7 ganglions and thoracic 1 ganglion, and its postganglionic nerve fibers are widely distributed in the area innervated by cervical 3 to thoracic 12 segments [9]. The anatomical position of the rat stellate ganglion is similar to that of humans. It is star-shaped or spindle-shaped. It starts from the dorsal side of the common carotid artery bifurcation, approximately at the level of C7 of the neck, with the subclavian vertebral arteries anterosuperior and the transverse process of C7 posteroinferiorly. Stellate ganglion block (SGB) is a commonly used nerve block technique in clinical practice. Local anesthetics are injected around the stellate ganglion, blocking the conduction of nerve impulses to the innervation area (head and face, upper limbs, chest, etc.). SGB was originally used to relieve cancer pain. With the continuous deepening of research, it has been found that SGB can not only act on the head and neck, upper chest, and upper limbs, but also the immune system, endocrine system, cardiovascular system, and so on [10]. A large number of studies have shown that SGB can block the preganglionic and postganglionic fibers of the sympathetic nerve, inhibit the excitatory conduction of it, and inhibit the vascular and glandular activities in its innervated areas; increase the blood flow of the innervated areas such as the head, face, and vertebrobasilar artery, improve tissue oxygen supply, and reduce the damage of oxygen-free radicals; block the excessive activation of the hypothalamus–pituitary–adrenal axis and inhibit the stress response [11, 12]. Studies have shown that SGB can reduce ALI caused by sepsis in a rat model [13]. Considering that both Dex and SGB can reduce ALI, combination medication may be a potential treatment approach for obesity-related ALI.

In this study, we established an ALI model in obese rats, combined SGB and Dex for the first time, and explored the effect on obesity-related ALI and its mechanism.

## 2. Materials and Methods

### 2.1. Experimental Animals

Thirty-six SPF grade 4-week-old male Wistar rats were bred in a 22°C, 50% relative humidity, 12 h/12 h light–dark cycle environment. All rats were fed a normal diet. After 7 days of adaptive breeding, follow-up experiments were carried out. The animal experiments described in this study were authorized by the Committee of Shanxi Bethune Hospital (SBQDL-2021-064).

### 2.2. Construction of the Obesity-Related ALI Model

After adaptive feeding, the rats were randomly divided into two groups: a normal diet group (control group, 6 rats) and a high-fat diet group (30 rats). They were fed continuously for 12 weeks, and the weights of the two groups of rats were measured and recorded every 3 weeks. After 12 weeks, an LPS-induced ALI model was used: 200 *μ*L of LPS (10 mg/mL, fully dissolved in 200 *μ*L of normal saline) was carefully instilled from the nostrils of the rat to allow the liquid to fully enter the rat's respiratory tract, and the rats were adjusted to a vertical position and rotated for 0.5–1 min to induce an ALI model with uniform distribution of LPS in the lungs. Rats in the normal control group were instilled with 200 *μ*L of normal saline via the nose in the same manner.

The rats were further divided into 6 groups, each with 6 rats: blank group (Control), normal diet rats were given 200 *μ*L normal saline via nasal drip; high-fat diet group (HFD), HFD rats were administered with 200 *μ*L normal saline via nasal drip; high-fat ALI model group (HFD + LPS), HFD rats were induced by 200 *μ*L LPS via nasal infusion; SGB group, HFD rats, the right SGB was treated with the cervical sympathetic trunk transection method, and 200 *μ*L LPS was instilled through the nose 30 minutes later; Dex group, rats on a high-fat diet, peritoneal injection of Dex (50 *μ*g/kg), 200 *μ*L LPS was injected through the nose 30 minutes later. SGB + Dex group, HFD rats, the right-side SGB was treated with cervical sympathetic trunk transection, and 50 *μ*g/kg Dex was injected intraperitoneally, and 200 *μ*L LPS was injected through the nose 30 minutes later. Twelve hours after modeling, blood was collected from the common carotid artery of the rats, and they were sacrificed by cervical dislocation to collect their lungs.

### 2.3. Stellate Ganglion Block

Intraperitoneal injection of the anesthetic (3% sodium pentobarbital 20 mg/kg) with a conventional anesthetic dose of about 2/3 was given to lightly anesthetize the rats. After the rat completed the step of stunning separation of the common carotid artery, the bifurcation of the common carotid artery was used as a mark, the spindle-shaped superior cervical ganglion on its dorsal side was found, and then a yellowish nerve conglomerate in the shape of a shuttle of about 2 mm was found from the origin of the vertebral artery or subclavian artery, which was the stellate ganglion, and the cervical sympathetic trunk was between the two ganglia. The carotid sympathetic trunk was disconnected, and the common carotid artery was ligated with 4.0 sutures. After disinfection, the incision was sutured layer by layer. If there are obvious symptoms of Honor syndrome, such as right pupil dilation, narrowed eye fissure, and ptosis after being awake lasting for more than 300 s, it indicates that the stellate ganglion model was successfully prepared [14].

### 2.4. Collection of Rat Bronchoalveolar Lavage Fluid (BALF)

After the rats were sacrificed, the neck was dissected, the trachea was exposed, the indwelling needle was inserted, fixed with a thin ligation and the needle core was pulled out, the syringe was attached, and the upper lobe of the right lung was lavaged with 0.5 mL PBS to obtain the BALF.

### 2.5. W/D Specific Gravity Method

After the rats were sacrificed, the lower lobe of the left lung was dissected, the blood on the surface of the lung tissue was blotted with filter paper, and the weight was weighed and recorded (labeled as wet weight: W). Thereafter, the samples were placed in an oven set at 60°C temperature and continuously baked for 48 h; the weight was weighed and recorded again (labeled as dry weight: D), and the W/D ratio of the lung tissue was calculated.

### 2.6. H&E Staining

After the rat lung tissue was fixed in 10% neutral formalin for 48 hours, the lung tissue was dehydrated with gradient alcohol, cleared with xylene, embedded in paraffin, and sectioned at 4 *μ*m thickness. After routine dehydration, the sections were stained with hematoxylin (Baoman Biological Co., Ltd., China) for 10 minutes, rinsed quickly with tap water for 30 s, separated with 1% hydrochloric acid alcohol for 1 minute, and rinsed for 1 minute. Then, they were stained with eosin and gradient alcohol dehydration (1 min/time). After xylene permeabilization, fixation with neutral resin was performed. Pictures were taken under an optical microscope and the morphology was observed. The lung tissue was scored from ranges 0 to 4 points: 0 points represent no damage or very slight damage; 1 point represents mild damage; 2 points represent moderate damage; 3 points represent severe damage; and 4 points represent extremely, severe damage [11].

### 2.7. TUNEL Staining

After gradient rehydration of the lung tissue sections, they were washed thrice with PBS for 5 min each time. 0.1% Triton X-100 was added to permeabilize the membrane for 20 minutes, and then transferred to 0.1% citric acid solution for 5 minutes. The sections were then washed thrice with PBS for 5 minutes each time. After air drying, 50 *μ*L of the TUNEL reaction mixture (Beyotime, Shanghai, China) was added and incubated for 1 h at 80% humidity and 37°C. After the incubation was completed, they were washed thrice with PBS, mounted with neutral resin, and observed and photographed under a confocal laser scanning microscope; the average number of TUNEL-positive cells (cell number in the field of view ≥30) were counted.

### 2.8. Detection of Biochemical Indicators

The lung tissue samples were thawed at room temperature; then, 30 mg of lung tissue was weighed, 400 *μ*L of lysate was added and cut in an EP tube with ophthalmic scissors, and then crushed with an ultrasonic homogenizer. Centrifugation at 12000 rpm at 4°C for 10 min was done and the supernatant was taken. According to the instructions of the corresponding kit (Beyotime), the activities of myeloperoxidase (MPO), superoxide dismutase (SOD), and glutathione peroxidase (GSH-Px) in the lung tissues of each group of rats were detected.

### 2.9. ELISA

The activities of TNF-*α*, IL-1*β*, and MCP1 in the rat alveolar lavage fluid of each group were detected according to the instructions of the corresponding ELISA kit (Multi sciences, China).

### 2.10. Western Blot

The lung tissue was lysed with RIPA Lysis Buffer (Beyotime), and the supernatant protein was obtained by centrifugation at 4°C, 12000 rpm for 15 min. After measuring the protein concentration with the BCA protein assay kit (Beyotime), the 20 *μ*g protein was separated using SDS-PAGE. Subsequently, the protein was transferred to the polyvinylidene difluoride (PVDF) membrane and placed in a blocking solution for 1 h at room temperature. Primary antibodies *β*-actin (4970, 1 : 1000, Cell Signaling, Boston, USA), glucose-regulated protein 78 (GRP78, #3183, 1 : 1000, Cell Signaling Technology, Boston, USA), C/EBP homologous protein (CHOP, #2895S, Cell Signaling Technology), protein kinase R-like endoplasmic reticulum kinase (PERK, #5683S, 1 : 1000, Cell Signaling Technology), and p-PERK (#3179S, 1 : 1000, Cell Signaling Technology) were added and incubated overnight at 4°C and shaken. After washing with PBST thrice the next day, 10 min each time, the secondary antibody was transferred (1 : 5000, Beijing Kangwei Century Biotechnology Co., Ltd., Beijing, China), incubated at room temperature for 1 h, and washed thrice after. After dripping the developing solution on the membrane, the chemiluminescence imaging system (Bio-rad) was used for detection.

### 2.11. Statistical Analysis

All experimental data were statistically analyzed by SPSS 22.0 software, and the data were expressed in the form of mean ± standard deviation (SD). The comparison between the two groups was analyzed by the *T*-test, and the comparison between multiple groups was analyzed by one-way analysis of variance. When *P* < 0.05, it represents that the difference in results was statistically significant. Graphpad Prism 8.0 (GraphPad Software, San Diego, CA, US) was used to graphically plot the data.

## 3. Results

### 3.1. SGB Combined with Dex Ameliorates Lung Tissue Damage in ALI Obese Rats

Firstly, the effect of SGB combined with Dex on ALI obese rats was tested. The results showed that after starting the high-fat diet, the weight of the rats in the HFD group was higher than that of the control group (Figure 1(a)), indicating that the obesity model was constructed. At the same time, compared with the control group, the water content of the lung tissue in the HFD + LPS group was significantly increased, while SGB and Dex could significantly reduce the water content of the lung tissue. In addition, it was lower after the combination of SGB and Dex (Figure 1(b)). H&E criteria for ALI include possible alveolar hemorrhage, lung cell necrosis, mild interstitial edema, and hyperplasia of connective tissue [15]. H&E staining was further used to observe the pathological structure of the lung tissue. The results showed that there was no obvious pathological damage in the control group, the alveolar structure was normal, the alveolar wall was intact, and there was no edema in the lumen. The lung tissue of the HFD group was hypertrophic compared to the normal group, little interstitial inflammatory cell infiltration was observed in the alveoli, there was no obvious congestion and hemorrhage, and the alveolar wall was intact. The alveolar wall in the lung tissue of the HFD + LPS group was destroyed, the alveolar wall was thickened with edema, and a collapse in the alveolar cavity was observed. A large number of inflammatory cell infiltration and red blood cell exudation could be observed in the alveolar walls and cavity in the lung tissues. Lung injury in the SGB, Dex, and SGB + Dex groups improved to varying degrees. The SGB + Dex group had the obvious improvement, and the increase in lung injury score was caused by the combination of HFD and LPS was significantly reduced (Figure 1(c)).

### 3.2. SGB Combined with Dex Can Reduce Cell Apoptosis and Inflammatory Response in Obese Rats with ALI

Further, through the detection of cell apoptosis and the release of inflammatory factors, the effect of SGB combined with Dex on obesity-related ALI was evaluated. The results showed that compared with the control group, the apoptosis rate of lung cells in the HFD group and the HFD + LPS group was significantly increased, while the use of SGB and Dex alone, as well as the combined use of SGB and Dex, could significantly inhibit lung cell apoptosis. At the same time, the effect of inhibiting cell apoptosis after SGB in combination with Dex was better than that of SGB and Dex alone (Figure 2(a)). Further inflammatory factor release results showed that compared with the control group, the levels of pro-inflammatory factors TNF-*α*, IL-1*β*, and MCP1 in the alveolar lavage fluid of the HFD + LPS group were significantly increased, while in the SGB, Dex, and SGB + Dex groups, TNF-*α*, IL-1*β*, and MCP1 levels were significantly reduced, and the SGB + Dex group had a better inhibitory effect on inflammatory factors (Figure 2(b)).

### 3.3. SGB Combined with Dex Reduces Oxidative Stress and Endoplasmic Reticulum Stress in ALI Obese Rats

On further examining the effects of SGB combined with Dex on oxidative stress and endoplasmic reticulum stress in obesity-related ALI rats, the results showed that HFD + LPS significantly increased the level of MPO in the lung tissue, and reduced the activity of SOD and GSH-Px, while the use of SGB and Dex alone or the combination of SGB and Dex significantly reduced the level of MPO in the lung tissue and increased the SOD and GSH-Px activity in the lung tissue, with the combination of SGB and Dex being more effective (Figure 3(a)). Further western blot detection results also showed that, compared with the control group, the protein expression levels of endoplasmic reticulum stress-related proteins GRP78, CHOP, and p-PERK in the lung tissue of the HFD + LPS group were significantly increased, and the p-PERK/PERK ratio was significantly increased. However, the protein expression levels of GRP78, CHOP, p-PERK, and p-PERK/PERK ratio in the lung tissues of the SGB, Dex, and SGB + Dex groups were significantly reduced. When the SGB + Dex group was compared with the SGB group and Dex group, the expression of endoplasmic reticulum stress-related proteins was lower (Figure 3(b)).

## 4. Discussion

Studies have shown that being overweight may affect the incidence and/or prognosis of ALI. It is estimated that about 20% of ICU patients are overweight or obese [16]. Biochemical changes in obese patients, such as increased inflammation and metabolic changes, may affect the risk of ALI in patients with other risk factors (such as sepsis) [17]. ALI is characterized by increased excessive lung inflammation [18], and inflammation plays an important role in the pathogenesis of ALI [19]. Studies have shown that SGB can inhibit the body's systemic inflammatory response by inhibiting the synthesis or secretion of pro-inflammatory cytokines such as IL-6, IL-10, and TNF-*α* [20]. Dex pretreatment can relieve pulmonary edema and hypertension in rabbits [21]. In addition, Dex can also reduce lung fibrosis in rats after ALI, and reduce the content of elastase that hydrolyzes lung tissue [22]. In the lungs, Dex can increase cGMP and prevent protein leakage from pulmonary vascular endothelial cells and pulmonary edema. In addition, recent studies have also found that Dex has a significant anti-inflammatory effect [23, 24]. In this study, it was found that both SGB and Dex alone can significantly reduce pulmonary edema, lung cell apoptosis, and the release of inflammatory factors TNF-*α*, IL-1*β*, and MCP1 in obese rats, and the combination of the two was more effective.

Myeloperoxidase (MPO) is a functional and activation marker of neutrophils, and its activity reflects the degree of neutrophil accumulation. The neutrophils that exist in the lung tissue can release a large amount of ROS and generate oxygen-free radicals themselves, ultimately leading to lung oxidative damage. At the same time, neutrophils themselves can release pro-inflammatory cytokines, which can aggravate the inflammatory response. Studies have shown that a core pathological feature of ALI is the accumulation of neutrophils and the increase of MPO activity [25]. If the accumulation of neutrophils in the lung is reduced, the severity of the lung injury can be significantly reduced [26]. SOD can decompose free radicals and protect healthy cells from those. Glutathione peroxidase (GSH-Px) is an important peroxide decomposing enzyme widely present in the body. In this study, it was also found that the combination of SGB and Dex can reduce the activity of MPO and up-regulate the activity of SOD and GSH-Px, suggesting that the combination of SGB and Dex can reduce oxidative stress and inhibit inflammation, thereby exerting lung protection.

Endoplasmic reticulum stress (ERS) is manifested by a large accumulation of misfolded and unfolded proteins in the lumen of the endoplasmic reticulum, impairing the normal physiological functions of the ER and triggering an unfolded protein response (UPR) [27]. A large number of studies have confirmed that there is oxidative stress damage in the pathogenesis of ALI, and the occurrence of oxidative stress in many diseases is mediated by ERS [28]. The PERK/CHOP signaling pathway is an important mechanism for ERS to mediate cell apoptosis [29]. GRP78, is a molecular chaperone protein connected to the unfolded protein under normal conditions, inhibits the activity of the latter, and plays an important role in maintaining endoplasmic reticulum homeostasis. When a misfolded protein accumulates in the endoplasmic reticulum, it can cause GRP78 to dissociate from the unfolded protein, activating them, and UPR occurs [30]. CHOP is another landmark protein of ERS, which is only expressed in a small amount in normal cells, and expressed in large amounts in ERS, which mediates the apoptosis pathway of the endoplasmic reticulum cells and eliminates damaged cells that cannot be repaired in time [31, 32]. In this study, it was found that the combination of SGB and Dex can reduce the protein expression levels of GRP78, CHOP, and p-PERK, indicating that the combination of SGB and Dex can exert a lung-protective effect on obesity-related ALI through the PERK/CHOP pathway.

## 5. Conclusion

In summary, the combined use of SGB and Dex can reduce obesity-related ALI, and its mechanism is related to reducing oxidative stress and endoplasmic reticulum stress, thereby inhibiting the release of inflammatory factors. This result can provide new directions and data support for the treatment of obesity-related ALI.

## Figures and Tables

**Figure 1:** The effect of SGB combined with Dex on ALI obese rats (a). Weight trend diagram of rats at 0, 3, 6, 9, and 12 weeks. (b) W/D specific gravity method detected the water content of rat lung tissue. (c) H&E staining showed the pathological damage of rat lung tissue in each group. ^*∗*^*P* < 0.05 and ^*∗∗*^*P* < 0.01*vs*. Control group; ^##^*P* < 0.01*vs.* HFD + LPS group; ^&&^*P* < 0.01*vs*. SGB group.

**Figure 2:** The effect of SGB combined with Dex on apoptosis and inflammation in obese rats with ALI (a). TUNEL staining detected the apoptosis of rat lung cells in each group. (b) ELISA detected the levels of TNF-*α*, IL-1*β*, and MCP1 in the alveolar lavage fluid. ^*∗*^*P* < 0.05, ^*∗∗*^*P* < 0.01, and ^*∗∗∗*^*P* < 0.001*vs*. Control group; ^##^*P* < 0.01 and ^###^*P* < 0.001*vs*. HFD + LPS group; ^&^*P* < 0.05*vs*. SGB group.

**Figure 3:** The effect of SGB combined with Dex on oxidative stress and endoplasmic reticulum stress in ALI obese rats. (a) Biochemical detection of the activities of MPO, SOD, and GSH-Px in the lung tissues of rats in each group. (b) Western Blot detection of the protein expression levels of GRP78, CHOP, PERK, and p-PERK in the lung tissues of rats; ^*∗*^*P* < 0.05 and ^*∗∗*^*P* < 0.01*vs*. Control group; ^##^*P* < 0.01*vs*. HFD + LPS group; ^&&^*P* < 0.01*vs*. SGB group.

## Data Availability

The data used to support the findings of this study are available from the corresponding author upon request.
